The article "MicroRNA-320a acts as a tumor suppressor by targeting BCR/ABL oncogene in chronic myeloid leukemia" was retracted in 2023. Reasons: duplicated images; duplicated text; signs of a paper mill; unreliable results or conclusions.

# MicroRNA-320a acts as a tumor suppressor by targeting BCR/ABL oncogene in chronic myeloid leukemia

**DOI:** 10.1038/srep12460

**Published:** 2015-07-31

**Authors:** Zhu Xishan, Lin Ziying, Du Jing, Liu Gang

**Affiliations:** 1 Clinical Research Center, Affiliated Hospital of Guangdong Medical College, 0086-027-7398722, China; 2 Weifang Traditional Chinese Medicine Hospital, Department of Urology. 0086-0536-8300338, China.

## Abstract

Accumulating evidences demonstrated that the induction of epithelial-mesenchymal transition (EMT) and aberrant expression of microRNAs (miRNAs) are associated with tumorigenesis, tumor progression, metastasis and relapse in cancers, including chronic myeloid leukemia (CML). We found that miR-320a expression was reduced in K562 and in CML cancer stem cells. Moreover, we found that miR-320a inhibited K562 cell migration, invasion, proliferation and promoted apoptosis by targeting BCR/ABL oncogene. As an upstream regulator of BCR/ABL, miR-320a directly targets BCR/ABL. The enhanced expression of miR-320a inhibited the phosphorylation of PI3K, AKT and NF-κB; however, the expression of phosphorylated PI3K, AKT and NF-κB were restored by the overexpression of BCR/ABL. In K562, infected with miR-320a or transfected with SiBCR/ABL, the protein levels of fibronectin, vimentin, and N-cadherin were decreased, but the expression of E-cadherin was increased. The expression of mesenchymal markers in miR-320a-expressing cells was restored to normal levels by the restoration of BCR/ABL expression. Generally speaking, miR-320a acts as a novel tumor suppressor gene in CML and miR-320a can decrease migratory, invasive, proliferative and apoptotic behaviors, as well as CML EMT, by attenuating the expression of BCR/ABL oncogene.

Chronic myeloid leukemia (CML) is a myeloproliferative disease originating from a constitutively active tyrosine kinase, BCR/ABL^1^. The BCR/ABL fusion protein is able to disorder the cell regulation system and confer malignant differentiation and proliferation of hematopoietic cells, thus directly contributing to leukemogenesis^2^. Therefore, formation of the BCR/ABL fusion gene is a key step in the pathogenesis of CML.

The treatment of CML has been greatly impacted by the development of imatinib which has been established as the standard therapy for CML^3^. While the hematopoietic stem cell (HSC) origin of CML was first suggested over 30 years ago, recently CML-initiating cells beyond HSCs are also being investigated. We have previously isolated fetal liver kinase-1-positive (Flk1^+^) mesenchymal stem cells (MSCs) carrying the BCR/ABL fusion gene from the bone marrow of Philadelphia chromosome-positive (Ph^+^) patients with hemangioblast property and they were proved to be the cancer stem cells in CML which differ from the normal MSCs^4^.

miRNAs are endogenously expressed, small noncoding RNAs that negatively regulate gene expression by causing degradation of target mRNAs, inhibition of the translation of these mRNAs or both^5^. miRNAs take a part in crucial cellular processes such as the stress response, development, differentiation, apoptosis, and proliferation^6^. Altered miRNA expression has been reported in numerous malignancies, including breast^7^, lung^8^, liver^9^, stomach^10^, colon^11^, brain^12^, leukemia^10^, and lymphoma^11^. An increasing number of studies have demonstrated that miRNAs can function as oncogenes or tumor suppressors, and they are often dysregulated in tumors^12^,^13^. So, oncogenic miRNAs are frequently upregulated, whereas tumor suppressing miRNAs are downregulated in tumors.

The article "MicroRNA-320a acts as a tumor suppressor by targeting BCR/ABL oncogene in chronic myeloid leukemia" was retracted in 2023. Reasons: duplicated images; duplicated text; signs of a paper mill; unreliable results or conclusions.

In the present study, we aimed to investigate the microRNAs that regulate BCR/ABL oncogene in CML and the possible mechanisms involved in this process. We examined miR-320a expression in 90 paired normal MSCs and CML cancer stem cells (BCR/ABL+ MSCs) by quantitative RT-PCR (qRT PCR) analysis. miR-320a was found to be strongly downregulated in CML cancer stem cells as compared with that of the normal MSCs. Moreover, decreased miR-320a was associated with poor prognosis and might independently predict overall survival (OS) and replase-free survival (RFS) in CML. Functional studies revealed that miR-320a suppressed K562 cell growth and metastasis by targeting BCR/ABL.

## Results

### The downregulation of miR-320a in K562

miRNA expression profiles of paired serum samples of CML patients before and after CRS (cytoreductive surgery) +HIPEC (intraperitoneal hyperthermic perfusion chemotherapy) were analyzed by miRCURY™ bead-based flow LNA microarray platform, using 5S RNA for normalization. The miRNA expression patterns differed significantly. Of the miRNAs assayed, miR-320a was down-regulated by more than 8-fold. MiR-320a expression was then evaluated by quantitative reverse transcription-PCR (qRT-PCR) in K562 and the normal control. The results indicated that miR-320a was significantly down-regulated in 4 CML cell lines compared with NC (Fig. 1A). Expressions of miR-320a were examined further by qRT-PCR in CML cancer stem cells and its matched normal MSCs from 70 CML patients (Fig. 1B). The results showed that the average expression level of miR-320a was significantly down-regulated in CML cancer stem cells compared to matched normal controls (Fig. 1C). Together these results provided strong evidence that miR-320a was significantly downregulated in CML. To further analyze the significance of miR-320a in terms of clinical prognosis, Kaplan-Meier survival analysis was performed using patient overall survival and relapse-free survival. The results demonstrated that patients with low miR-320a expression had shorter median OS and RFS than did patients with high miR-320a expression (Fig. 1D).

The article "MicroRNA-320a acts as a tumor suppressor by targeting BCR/ABL oncogene in chronic myeloid leukemia" was retracted in 2023. Reasons: duplicated images; duplicated text; signs of a paper mill; unreliable results or conclusions.

### MiR-320a inhibits K562 migration, invasion, proliferation and induces apoptosis by BCR/ABL

To examine the functional significance of miR-320a overexpression in K562, we infected the CML cell line K562 with LV-hsa-miR-320a. Compared with the expression of cont-miR, miR-320a was significantly overexpressed in the K562 after infection with LV-hsa-miR-320a (Fig. 2A). We also found that, comparing with cont-miR, the expression of BCR/ABL was significantly downregulated in the K562 cell lines after infection with LV-hsa-miR-320a (Fig. 2B). The cells with forced expression of miR-320a exhibited significantly decreased proliferation compared with the cells with forced expression of cont-miR (Fig. 2C). The miR-320a-infected cells also exhibited reduced colony formation ability: the number of foci in the miR-320a-expressing cells was decreased compared with the cont-miR-infected cells (Fig. 2D). miR-320a could regulate the expression of BCR/ABL by directly inhibiting BCR/ABL transcript or other indirect circuits, so we next ascertained whether the reduction of BCR/ABL expression could explain the inhibition of CML cell migration, invasion and proliferation observed after the forced expression of miR-320a. We therefore forced the expression of miR-320a in K562 cells together with a construct containing the BCR/ABL coding sequence but lacking the 3′UTR of the BCR/ABL mRNA. As a result, this construct yielded a BCR/ABL mRNA that was resistant to miR-320a. We found that CML cell migration, invasion, proliferation and apoptosis were restored in the K562 cell line with forced miR-320a expression and BCR/ABL restoration (Fig. 2E–G). Those results show that miR-320a inhibits CML cell migration, invasion and proliferation and promotes apoptosis by targeting its BCR/ABL oncogene.

### Overexpression of miR-320a prohibits tumorigenesis and promotes apoptosis *in vivo*

We next examined whether overexpression of miR-320a could suppress tumor growth and induce apoptosis *in vivo*. Retrovirus-mediated K562/miR-320a and K562/miR-control stable cell lines were obtained as described in the retroviral transfection for stable cell lines section. RV-miR-320a, RV-miR-control or K562 cells were injected subcutaneously into nude mice, and tumor formation was monitored. After 35 days, the mice were euthanized and tumor weights were measured. Tumors grew faster in RV-miR-control and parental cell K562 group than that in the group of RV-miR-320a (Fig. 3A–D). The average weight of tumors resulting from RV-miR-320a was significantly less than tumors derived from RV-miR-control or K562 cells (670 ± 130 mg vs. 1810 ± 420 mg, 1980 ± 220 mg; p < 0.01). There was no significant difference in the tumor volume or in the weight between RV-miR-control or K562 cells.

The article "MicroRNA-320a acts as a tumor suppressor by targeting BCR/ABL oncogene in chronic myeloid leukemia" was retracted in 2023. Reasons: duplicated images; duplicated text; signs of a paper mill; unreliable results or conclusions.

In addition, the number of Ki-67-antigen-positive cells was lower in the tumor derived from RV-miR-320a cells than that in RV-miR-control or K562 cells (p < 0.01, Fig. 3E). The results revealed that the decreased tumor growth in mice was, in part, due to lower proliferation caused by the overexpression of miR-320a. Thus, tumorigenicity was significantly reduced in RV-miR-320a cells *in vivo*. To assess whether tumor growth inhibition in RV-miR-320a was due partly to the induction of apoptosis partly, TUNEL assays of tumor tissues were performed. As shown in Fig. 3E, the RVmiR-320a cells showed a more tumor cell positive staining and a significantly higher apoptotic index than the K562/vector or K562 cells (P < 0.01). These results suggested that miR-320a inhibition of tumorigenicity was attributed to decreased proliferation and increased apoptosis *in vivo*.

### miR-320a directly targets and inhibits BCR/ABL

To understand how miR-320a suppress CML growth and metastasis, we used three algorithms (Targetscan, Pictar and Miranda) to help identify miR-320a targets in human CML. Of these target genes that were predicted by all three algorithms, BCR/ABL attracted our attention immediately as it has been implicated in tumorigenesis or metastasis and proved to be the oncogene previously.

We cloned the full-length BCR/ABL 3′-UTR into a luciferase reporter vector. Luciferase assay revealed that miR-320a directly bound to BCR/ABL 3′-UTR, and by which it remarkably reduced luciferase activities (Fig. 4A). However, mutation of the putative miR-320a sites in the 3′-UTR of BCR/ABL abrogated luciferase responsiveness to miR-320a (Fig. 4A). To directly assess the effect of miR-320a on BCR/ABL expression, we performed western blot analysis. As seen in Fig. 4B, lentiviral induced ectopic miR-320a dramatically suppressed the BCR/ABL protein levels in K562 cells. Furthermore, knockdown of miR-320a, through transfection of anti-miR-320a, in A562 cells increased BCR/ABL protein levels (Fig. 4B). Taken together, these results indicate that BCR/ABL is a direct downstream target for miR-320a in CML cells. To further elucidate the relationship between miR-320a and BCR/ABL expression in primary samples, we did the scatter plot and the Pearson correlation analysis, the results indicated that miR-320a expression was negatively correlated with the target protein levels in the CML samples (Fig. 4C).

The article "MicroRNA-320a acts as a tumor suppressor by targeting BCR/ABL oncogene in chronic myeloid leukemia" was retracted in 2023. Reasons: duplicated images; duplicated text; signs of a paper mill; unreliable results or conclusions.

The above results prompted us to examine whether miR-320a suppresses CML growth and metastasis through repressing BCR/ABL expression. For this purpose, BCR/ABL was re-expressed in miR-320a transfected K562 cells. In miR-320a-expressing cells, re-expression of BCR/ABL rescued the invasion and growth defects of miR-320a (Fig. 4D–F). Finally, we tested if miR-320a expression correlated with BCR/ABL protein levels in CML. There was an inverse correlation between the BCR/ABL protein levels, indicated by immunohistochemistry staining, and miR-320a expression assessed by *in situ* hybridization in 90 CML cancer stem cells on TMAs as used above (Fig. 4G).

### MiR-320a regulates CML pathogenesis by targeting BCR/ABL induced PI3K/AKT/ NF-κB signaling pathways

CML is a clonal hematopoietic stem cell disorder characterized by the t (9;22) chromosome translocation and resultant production of the constitutively activated BCR/ABL tyrosine kinase and it has been proved to be the tumor oncogene. PI3K signaling pathway was indicated to be induced by BCR/ABL by our past study. Because BCR/ABL is a downstream target of miR-320a, we assumed that miR-320a could decrease the expression of the phosphorylation of PI3K, AKT, and NF-κB. We found that the forced expression of miR-320a inhibited the phosphorylation of PI3K, but the relative expression level of total PI3K was not significantly altered. miR-320a could also decrease the phosphorylation of AKT and NF-κB (Fig. 5A). miR-320a could bind the 3′UTR of the BCR/ABL mRNA to regulate the phosphorylation of PI3K, AKT and NF-κB; however, we did not know whether miR-320a could bind the 3′ UTRs of other genes to achieve an equal effect. So rescue experiment was performed, and the restoration of BCR/ABL expression was confirmed through an immunoblot analysis (Fig. 5B). We found that the phosphorylation levels of PI3K, AKT and NF-κB were not significantly altered in the K562 cells with forced miR-320a expression and BCR/ABL restoration (Fig. 5C). Therefore, we conclude that miR-320a regulates the phosphorylation of PI3K, AKT and NF-κB via BCR/ABL.

### MiR-320a controls the epithelial phenotype of CML

EMT is an important mechanism associated with cancer invasiveness and metastasis. The phenomenon of EMT is defined as the transition of epithelial cells to fibroblastoid- or mesenchymal-like cells. EMT is characterized by the loss of epithelial markers and the acquisition of mesenchymal components. Ecadherin, occludin and cytokeratin are downregulated during EMT, whereas N-cadherin, vimentin and fibronectin are upregulated. To find the role of BCR/ABL in sustaining the mesenchymal phenotype of CML cells, we knocked down the expression of BCR/ABL by RNA interference (RNAi) (Fig. 6A) and examined the expression of mesenchymal markers such as fibronectin, N-cadherin E-cadherin and vimentin in K562 cells. We found that the expression levels of fibronectin, vimentin and N-cadherin were decreased but the expression of E-cadherin was increased in the BCR/ABL-depleted tumor stem cells (Fig. 6B). The result shows that BCR/ABL can drive EMT process in CML. Because BCR/ABL is a downstream target of miR-320a, we assumed that miR-320a could determine the epithelial phenotype of CML. To determine whether the molecular changes typical of a reduced EMT occurred in miR-320a-expressing cells, we examined the expression of mesenchymal and epithelial markers in K562. The immunoblot analysis showed that the expression levels of fibronectin, vimentin and N-cadherin were decreased in the K562 with the forced expression of miR-320a. Furthermore, the forced expression of miR-320a increased the expression of E-cadherin in the K562 cell line, whereas the control-infected cells remained E-cadherin negative. We found that miR-320a regulated the phosphorylation of PI3K, AKT and NF-κB via BCR/ABL; therefore, we detected whether miR-320a could regulate EMT via BCR/ABL. The immunoblot analysis showed that the expression of the above mesenchymal markers in the miR-320a-expressing cells was restored to the normal level by the restoration of BCR/ABL expression (Fig. 6C). Altogether, these results demonstrated that miR-320a could inhibit EMT via BCR/ABL in CML.

The article "MicroRNA-320a acts as a tumor suppressor by targeting BCR/ABL oncogene in chronic myeloid leukemia" was retracted in 2023. Reasons: duplicated images; duplicated text; signs of a paper mill; unreliable results or conclusions.

## Discussion

Expression of the Philadelphia chromosome (Ph), the t (9;22) chromosomal translocation and the formation of the BCR/ABL fusion protein, is the hallmark of chronic myeloid leukemia (CML)^14^,^15^. The BCR/ABL1 oncogene contributes to the development of CML clones^16^. Although Interferon-α, Imatinib (a BCR/ABL tyrosine kinase inhibitor) and stem cell transplantations are the standard therapeutic options, transplant-related morbidity from graft-versus-host disease and mortality rates of 10% to 20% have greatly reduced the allogeneic hematopoietic cell transplantation in clinics, while interferon-α is only effective in some patients to some degree and chemotherapeutic intervention does not result in prolonged overall survival and the reason is possibly due to some unknown biology of the CML cancer stem cells especially the regulating molecule mechanisms^17^,^18^,^19^.

Our laboratory have identified the Flk-1 +CD34-CD31- hemangioblasts as the CML initiating cells and proved the rearrangement of the BCR/ABL gene might happen at the level of this hemangioblastic progenitor cells instead of HSCs^20^. Based on this concept, we first used qRT-PCR and ISH to show that miR-320a levels in CML cancer stem cells were significantly lower than the normal MSCs in healthy donors. Moreover, the miR-320a levels were associated with the clinical stage and presence of lymph node metastases. Kaplan-Meier survival analysis revealed that patients whose MSCs displayed low expression of miR-320a had a shorter OS and RFS in CML. In addition, Cox proportional hazards regression analysis showed that reduced miR-320a in CML was a strong and independent predictor of shorter OS and RFS. Moreover, the overexpressed miR-320a could inhibit K562 cell migration, invasion and proliferation, and promote apoptosis. Meanwhile, those tumourigenic qualities can be completely restored by BCR/ABL overexpression. In addition, the luciferase reporter assays suggested that miR-320a targets BCR/ABL oncogene directly. Thus, we conclude that miR-320a acts as a potential tumor suppressor in CML, a function that is accomplished by curbing the expression of BCR/ABL.

The article "MicroRNA-320a acts as a tumor suppressor by targeting BCR/ABL oncogene in chronic myeloid leukemia" was retracted in 2023. Reasons: duplicated images; duplicated text; signs of a paper mill; unreliable results or conclusions.

As an oncogene, BCR/ABL played important roles in the pathogenesis in CML^21^,^22^,^23^,^24^. More and more signaling pathways were proved to be involved in the regulation of BCR/ABL on CML^25^,^26^,^27^. In this study, we found that overexpressed miR-320a could decrease the expression of the phosphorylation of PI3K, AKT and NF-κB, an effect that was reversed upon BCR/ABL restoration. The activation of PI3K, AKT and NF-κB in association with apoptosis resistance/cell survival has been well documented in a variety of model systems^28^,^29^,^30^. Thus, we conclude that miR-320a inhibits CML cell migration, invasion and proliferation, as well as promoting apoptosis, by decreasing the expression of BCR/ABL, which increases PI3K, AKT and NF-κB signaling.

The phenotypic transition from an epithelial to a mesenchymal like cell state represents an important mechanism of epithelial plasticity and cancer metastasis^31^,^32^,^33^. MicroRNAs have recently emerged as potent regulators of EMT due to their ability to target multiple components involved in epithelial integrity or mesenchymal traits. The miR-200 family has been shown to directly target EMT transcription factor families^34^. In human mammary epithelial cells, miR-9 directly targets E-cadherin, thus promoting the mesenchymal phenotype, including increased cell migration and invasion^35^. MiR-27 promotes human gastric cancer cell metastasis by inducing the epithelial-to-mesenchymal transition^36^. We thereby performed the assay that tested the relationships between miR-320a and EMT, and our *in vitro* experiments strongly demonstrated that miR-320a promote EMT of CML. Furthermore, we found higher phosphorylation of PI3K, AKT and NF-κB when we test the EMT hallmark N-cadherin, vimentin, fibronectin and E-cadherin of K562 transfected with miR-320a. Interestingly, blocking the PI3K/AKT/NF-κB pathway cancelled the effect of miR-320a, which might provide a more comprehensive picture of the molecular network that miR-320a promoted EMT through activating PI3K/AKT/NF-κB pathway in metastasis of CML.

The article "MicroRNA-320a acts as a tumor suppressor by targeting BCR/ABL oncogene in chronic myeloid leukemia" was retracted in 2023. Reasons: duplicated images; duplicated text; signs of a paper mill; unreliable results or conclusions.

## Material and Methods

### Patient samples

90 patients with newly diagnosed CML (49 male and 41 female, aged 17-71 years) were recruited in this study. All were Ph^+^ patients with CML in chronic phase as revealed by bone marrow histology and cytogenetic analysis and the immunophenotypes of thawed cells were quite variable. None was treated with hydroxyurea or interferon before. The control samples were from 90 healthy donors (48 male and 42 female, aged 19-68 years). They were all Ph^+^ negative at donation. Bone marrow samples were collected after obtaining informed consent according to procedures approved by the Ethics Committee at the Institute of the 309^th^ hospital of People’s Liberation Army.

### Cell preparations and culture conditions

Isolation and culture of bone marrow-derived BCR/ABL^+^ MSCs from CML patients were performed as described previously with some modifications^19^,^20^,^21^. Briefly, mononuclear cells were separated by a Ficoll-Paque gradient centrifugation (specific gravity 1.077 g/mL; Nycomed Pharma AS, Oslo, Norway) and the sorted cells were plated at concentration of 1 cell/well by limiting dilution in a total of 96 × 10 wells coated with fibronectin (Sigma, St Louis, MO) and collagen (Sigma) for each patient. Culture medium was Dulbecco modified Eagle medium and Ham F12 medium (DF12) containing 40% MCDB-201 medium complete with trace elements (MCDB) (Sigma), 2% fetal calf serum (FCS; Gibco Life Technologies, Paisley, United Kingdom), 1 × insulin transferrin selenium (Gibco Life Technologies), 10^−9^ M dexamethasone (Sigma), 10^−4^ M ascorbic acid 2-phosphate (Sigma), 20 ng/mL interleukin-6 (Sigma), 10 ng/mL epidermal growth factor (Sigma), 10 ng/mL platelet-derived growth factor BB (Sigma), 50 ng/mL fetal liver tyrosine kinase 3 (Flt-3) ligand (Sigma), 30 ng/mL bone morphogenetic protein-4 (Sigma), 100 U/mL penicillin and 100 ug/mL streptomycin (Gibco Life Technologies) at 37 °C and a 5% CO_2_ humidified atmosphere. Culture media were changed every 4 to 6 days.

### RT-PCR

RNA isolation and reverse transcription were performed as previously described^32^. Oligonucleotide primer sequences were as follows: β-actin (264 bp), forward: 5′-GAG ACC TTC AAC ACC CCA GCC-3′; reverse:5′-AAT GTC ACG CAC GAT TTC CC-3′; BCR/ABL (271 bp), forward: 5′-AGA GGT CTC AGA AGG GAC CG-3′, reverse: 5′-GGG CCA TAC AGG ACA CGA AG-3′; PI3K (174 bp), forward: 5′-TGC TTT TTC CAG GGG TGT GTT-3′, reverse: 5′-TAC TTC CTG CAC TAA TTT GGC A-3′; AKT (201 bp), forward: 5′-GGA AAC CCA CAA CGA AAT CTA TGA C-3′, reverse: 5′-TTG CTG AGG TAT CGC CAG GAA T-3′; NF-κB (225 bp), forward: 5′-CGC CAA GGA GGT TTA CAA AAT AGA C-3′, reverse: 5′-TCA ATC CGT TGT TCA GGC ACT CT-3′. For all the above genes, amplification was performed under the same cycling conditions (1 minute at 94 °C, 50 seconds at 57 °C, 1 minute at 72 °C), except the number of cycles that were specified for each gene (31 for BCR/ABL  `  PI3K and AKT, 32 for NF-κB).

The article "MicroRNA-320a acts as a tumor suppressor by targeting BCR/ABL oncogene in chronic myeloid leukemia" was retracted in 2023. Reasons: duplicated images; duplicated text; signs of a paper mill; unreliable results or conclusions.

### Western blot and Immunopreciptation

MSCs were harvested at specific times after treatment with reagents as indicated in each experiment. Cells were mixed with loading buffer and subjected to electrophoresis. After electrophoresis proteins were transferred to polyvinyl difluoride membranes (Pall Filtron) using a semidry blotting apparatus (Pharmacia) and probed with mouse monoclonal antibodies, followed by incubation with peroxidase-labeled secondary antibodies. Detection was performed by the use of a chemiluminescence system (Amersham) according to the manufacturer’s instructions. Then membrane was striped with elution buffer and reprobed with antibodies against the nonphosphorylated protein as a measure of equal loading. Controls for the immunoprecipitation used the same procedure, except agarose beads contained only mouse IgG.

### RNA-i experiments

The si-RNA sequence targeting human BCR/ABL (from mRNA sequence; Invitrogen online) corresponds to the coding region 286–314 relative to the first nucleotide of the start codon (target = 5′-ATC TTC ACT CAA TAG GTA CGA ACG GC-3′). Computer analysis using the software developed by Ambion Inc. confirmed this sequence to be a good target. si-RNAs were 21 nucleotides long with symmetric 2-nucleotide 3′ overhangs composed of 2′-deoxythymidine to enhance nuclease resistance. The si-RNAs were synthesized chemically and high pressure liquid chromatography purified (Genset, Paris, France). Sense si-RNA sequence was 5′-UAC TAC CAA AUG UAT CCT AdTdT-3′. Antisense si-RNA was 5′-AUG AAT CTA AUC GTU GAA GdTdA-3′. For annealing of si-RNAs, mixture of complementary single stranded RNAs (at equimolar concentration) was incubated in annealing buffer (20 mM Tris-HCl pH 7.5, 50 mM NaCl, and 10 mM MgCl_2_) for 2 minutes at 95 °C followed by a slow cooling to room temperature (at least 25 °C) and then proceeded to storage temperature of 4 °C. Before transfection, cells cultured at 50% confluence in 6-well plates (10 cm^2^) were washed two times with OPTIMEM 1 (Invitrogen) without FCS and incubated in 1.5 ml of this medium without FCS for 1 hour. Then, cells were transfected with BCR/ABL-RNA duplex formulated into Mirus *Trans*IT-TKO transfection reagent (Mirus Corp, Interchim, France) according to the manufacturer’s instructions. Unless otherwise described, transfection used 20 nM RNA duplex in 0.5 ml of transfection medium OPTIMEM 1 without FCS per 5 × 10^5^ cells for 6 hours and then the medium volume was adjusted to 1.5 ml per well with RPMI 2% FCS. SilencerTM negative control 1 si-RNA (Ambion Inc.) was used as negative control under similar conditions (20 nM). The efficiency of silencing is 80% in our assay.

The article "MicroRNA-320a acts as a tumor suppressor by targeting BCR/ABL oncogene in chronic myeloid leukemia" was retracted in 2023. Reasons: duplicated images; duplicated text; signs of a paper mill; unreliable results or conclusions.

### Migration and invasion assays

We used a Transwell insert (24-well insert, pore size 8 lm; Corning, Inc., Corning, NY) to determine the effect of miR-320a on K562 migration and invasion *in vitro*. Briefly, the transfected cells were first starved in serum-free medium overnight, and 3 × 10^4^ cells were re-suspended in serum-free medium and placed in the top chambers in triplicate. The lower chamber was filled with 10% FBS as the chemo-attractant and incubated for 48 h for the migration assay and 72 h for the invasion assay. For the invasion assay, the inserts were previously coated with extracellular matrix gel (BD Biosciences, Bedford, MA). At the end of the experiments, the cells on the upper surface of the membrane were removed, and the cells on the lower surface were fixed and stained with 0.1% crystal violet. Five visual fields of each insert were randomly chosen and counted under a light microscope.

### Colony formation assay

Six-well plates were covered with a layer of 0.6% agar in medium supplemented with 20% fetal bovine serum. Cells were prepared in 0.3% agar and seeded in triplicate. After the plates were incubated at 37□ for two weeks, the colonies were counted.

### Apoptosis analysis

The apoptotic cells were evaluated by Annexin V-FITC and propidium iodine staining (BD, USA) and analyzed with a FACS Calibur instrument (BD, USA). The collected data were analyzed using flow soft ware.

### Tumor-bearing (Xenografts) study

As reported recently^7^, 1.5 × 10^5^ K562 cells re-suspended in 150 ul PBS were injected subcutaneously into the flank of the normal C57B/l6 mice at age about 8 weeks (5 mice per group). Both K562 and the mice were in C57BL/6 background and no rejection occurred. The animals were maintained in a pathogen-free barrier facility and closely monitored by animal facility staff. The grown tumors (xenografts) were measured every 3 day starting 23 days post inoculation of cells using caliper as length × width × width/2 (mm^3^). 6.3 ug of miR-320a precursor or negative miRNA (GenePharma, Shanghai, China) mixed with 1.6 ul transfection reagent Lipofectamine 2000 (Invitrogen) in 50 ul PBS were injected into the tumors every 3 days, for total of 3 times. 32 days after inoculation, the animals were sacrificed and the xenografts were isolated, the weight (gram) and volume (mm^3^) of the xenografts were determined. All procedures were conducted according to the Animal Care and Use guideline approved by Xinxiang Medical University Animal Care Committee.

The article "MicroRNA-320a acts as a tumor suppressor by targeting BCR/ABL oncogene in chronic myeloid leukemia" was retracted in 2023. Reasons: duplicated images; duplicated text; signs of a paper mill; unreliable results or conclusions.

### Statistical Analysis

Student’s t-test (two-tailed), One-way ANOVA and Mann-Whitney test were employed to analyze the *in vitro* and *in vivo* data using SPSS 12.0 software (Chicago, IL, USA). P value < 0.05 was defined as statistically significant.

## Additional Information

**How to cite this article**: Xishan, Z. *et al*. MicroRNA-320a acts as a tumor suppressor by targeting BCR/ABL oncogene in chronic myeloid leukemia. *Sci. Rep*. **5**, 12460; doi: 10.1038/srep12460 (2015).

## Figures and Tables

**Figure 1:** Downregulation of miR-320a expression in CML cell lines and CML cancer stem cells compared with the corresponding controls. (**A**). Relative expression of miR-320a in 4 CML cell lines and one normal control were detected by qRT-PCR. All experiments were repeated at least three times. Each bar represents the mean of three independent experiments. *P < 0.05. (**B**). Relative expression of miR-320a in 70 specimens of CML cancer stem cells and normal MSCs were carried out by qRT-PCR. Data are shown as –△△CT values. (**C**) The mean and standard deviation of miR-320a expression levels in 70 specimens of CML cancer stem cells and normal MSCs were shown. Data are presented as 2^−△Ct^ values (**P < 0.01). (**D**). Survival analysis of CML. OS and RFS curves for 90 CML patients with high or low miR-320a expression were constructed using the Kaplan-Meier method and evaluated using the log-rank test.

**Figure 2:** miR-320a inhibits CML cell migration, invasion, proliferation and induces apoptosis. (**A**) The miR-320a expression was significantly increased in K562 after infection with LV-hsa-miR-320a. (**B**) The BCR/ABL expression was significantly decreased in K562 after infection with LV-hsa-miR-320a. (**C**) K562 proliferation was significantly reduced after LV-hsa-miR-320a infection compared with cont-miR infection. (**D**) miR-320a overexpression significantly inhibited the colony-forming ability of K562. (**E**–**G**) K562 cell migration, invasion, proliferation and apoptosis were restored after BCR/ABL restoration. The data represent the means ± s.d.; *p < 0.001, **p < 0.05, ***p < 0.01.

The article "MicroRNA-320a acts as a tumor suppressor by targeting BCR/ABL oncogene in chronic myeloid leukemia" was retracted in 2023. Reasons: duplicated images; duplicated text; signs of a paper mill; unreliable results or conclusions.

**Figure 3:** Overexpression of miR-320a inhibits tumorigenicity and increases apoptosis *in vivo*. (**A**) Photographs of tumors derived from RV-miR-320a, RV-miR-control or K562 cells in nude mice. (**B**) Growth kinetics of tumors in nude mice. Tumor diameters were measured every 7 days. (*p < 0.05, **p < 0.01).(**C**) Average weight of tumors in nude mice. (**p < 0.01). (**D**) Comparison of proliferation index. (*p < 0.05). (**E**) The percentage of apoptotic cells was counted. (**p < 0.01).

**Figure 4:** miR-320a directly targets BCR/ABL. (**A**) The 3′-UTR element of BCR/ABL messenger RNA was partially complementary to miR-320a. miR-320a, anti-miR-320a or scramble control and luciferase reporter containing either a wild type or a mutant 3′-UTR were co-transfected into HEK-293T cells. And a Renilla luciferase expressing construct exerts as internal control. (**B**) Western blot analysis of BCR/ABL expression in K562 cells infected with miR-320a, and NC transfected with miR-320a inhibitors (Anti-miR-320a). The gels have been run under the same experimental conditions. (**C**). Analysis of correlation of miR-320a and BCR/ABL expression in CML cancer stem cells and normal MSCs. *p < 0.05, **p < 0.01, ***p < 0.001. The analysis indicated that BCR/ABL and miR-320a were negatively correlated. (**D**–**F**) BCR/ABL abrogated the suppressive roles of miR-320a in K562 invasion and growth. K562 cells stably expressing miR-320a or scramble were transfect with or without BCR/ABL plasmids. Invasion assays (**D**), apoptosis analysis (**E**) and cell proliferation analysis (**F**) were performed with the above cells as described in Materials and Methods. Data are presented as mean ± s.e.m from at least three independent experiments. (**G**) Spearman’s correlation scatter plot of the levels of miR-320a (determined by *in situ* hybridization) and BCR/ABL protein (determined by immunohistochemistry) in 90 CML specimens. Representative images of BCR/ABL expression by immunohistochemistry were shown. Original magnification: ×200.

**Figure 5:** miR-320a down-regulates the phosphorylation of PI3K, AKT and NF-κB via BCR/ABL. (**A**) The phosphorylation and total expression levels of PI3K, AKT and NF-κB in K562 cells infected with LV-hsa-miR-320a or cont-miR. (**B**) An immunoblot analysis of BCR/ABL expression in K562 cells infected with LV-hsa-miR-320a or cont-miR, with or without BCR/ABL restoration. (**C**) The phosphorylation and total expression levels of PI3K, AKT and NF-κB in K562 cells infected with LV-hsa-miR-320a or cont-miR, with or without BCR/ABL restoration. The expression levels of the phosphorylated proteins were normalized to those of the respective total proteins. The data represent the means ± s.d.; *p < 0.01. All the gels have been run under the same experimental conditions.

The article "MicroRNA-320a acts as a tumor suppressor by targeting BCR/ABL oncogene in chronic myeloid leukemia" was retracted in 2023. Reasons: duplicated images; duplicated text; signs of a paper mill; unreliable results or conclusions.

**Figure 6:** miR-320a promotes an epithelial phenotype in K562. (**A**) Right panel: BCR/ABL expression was detected by western blot in K562 cells after treatment with 3 independent siRNA sequences (siNRP1) or a control (siC). Left panel: Relative expression of BCR/ABL was shown in the histogram. (**B**) Right panel: An immunoblot analysis of N-cadherin, vimentin, fibronectin and E-cadherin in K562 cells transfected with siNRP1 or siC. Left panel: Relative expression of proteins was shown in the histogram. (**C**) An immunoblot analysis of N-cadherin, vimentin, fibronectin and Ecadherin in K562 cells infected with LV-hsa-miR-320a or cont-miR, with or without BCR/ABL restoration. The protein expression levels were normalized to Actin. The data represent the means ± s.d.; *p < 0.01. All the gels have been run under the same experimental conditions.
